RETRACTED

# A Study on the Strategy of Sustainable Governance of NIMBY Movements: Focusing on Civil Environmental Rights

**DOI:** 10.1155/2022/2514373

**Published:** 2022-08-25

**Authors:** Chen Cao

**Affiliations:** Law School, Xiangtan University, Xiangtan 411105, Hunan, China

## Abstract

It is a common problem faced by countries in the process of industrialization and urbanization that citizens oppose the construction of negative externality facilities near their residence. Environmental right is one of the basic rights enjoyed by citizens and also an important part of human rights, allowing citizens to participate in their own environmental use decisions and defend their own environmental rights and interests against infringement. This paper focuses on the basic environmental rights of citizens, essentially defines the NIMBY movement as a movement for justice in which citizens advocate for equal environmental rights and interests, and analyzes the movement's rationale or the fundamental environmental rights of citizens. Disregard for citizens' substantive and procedural environmental rights and interests is linked to NIMBY movements. At the same time, compared with the traditional campaign-styled governance paradigm, the sustainable development governance emphasizes joint negotiation and multiple interactions, which can better maximize the environmental benefits of the whole governance cycle. Therefore, this paper discussed the governance path of NIMBY from two dimensions: determining the boundaries of citizens' substantive environmental rights and interests for enhancing their sense of identity and protecting citizens' procedural environmental rights and interests by laying more emphasis on the sustainable governance of NIMBY movements.

## 1. Introduction

Currently, NIMBY incidents occur from time to time, while the solution is often limited by the pressure of maintaining stability and the dilemma characterized by protest, compromise, and construction suspension. The limitations are attributed to the failure to adopt a strategy of sustainable governance. A NIMBY movement may be perceived as socially destabilizing and met with rude suppression or a compromise when suppression fails, leading to a bizarre circle of “distribution by the degree of instability.” In turn, such a situation radicalizes a NIMBY movement. Since the NIMBY itself is a product of unequal distribution of citizens' environmental rights and interests, it is particularly important to explore NIMBY movements by focusing on citizens' basic environmental rights, analyze the nature and causes of NIMBY movements, and discuss the path of sustainable governance in a bid to solve the NIMBY dilemma. Meanwhile, sustainable development governance refers to the rule of law process in which the government, the market, enterprises, social organizations, and the public jointly manage public affairs and assume public responsibilities through joint consultation and other interactive ways based on their common rights, so as to continuously maximize public interests and maintain social justice [1]. The nature of the NIMBY movement determines that it needs to be governed by sharing rights and jointly negotiating in order to maximize the governance efficiency.

RETRACTED

## 2. Civil Environmental Rights: A Focus on Exploring NIMBY Movements

### 2.1. NIMBY and Civil Environmental Rights

Not in My Backyard (NIMBY), a term first proposed by O'Hare in his paper, refers to the opposition of citizens to public facilities being built in their neighborhood. NIMBY movement means that citizens fear some construction projects (toxic waste disposal sites or landfills, incineration sites, etc.) which may have negative impacts on the quality of the surrounding environment, asset value, or physical and mental health, which in turn breeds aversion and antagonistic behavior [2]. Since the waste incineration power generation project in Liulitun, Haidian District, Beijing, was protested by residents in 2006, the conflicts caused by the construction of waste treatment facilities have occurred from time to time, resulting in great impact. For example, due to the government's late publicity of the information on the waste incineration power generation project before the project approval in Yuhang District of Hangzhou, the surrounding public lacked understanding of the project construction information, which led to the emergence of a large-scale neighborhood avoidance movement. For another example, due to the failure to publicize the kitchen waste resource treatment station project in Xi'erqi, Haidian District, Beijing, residents believed that the site selection of the project was unreasonable, because there were many residential quarters, kindergartens, primary and secondary schools, hospitals, and other public institutions around the project, which lead to large-scale petitions [3]. By the degree of citizens' resistance, NIMBY movements can be roughly divided into the pre-NIMBY period when citizens lack knowledge of toxic pollutants, the early NIMBY period when discrete sporadic resistance is done, and the post-Love Canal period when aggregated resistance occurs. The research on NIMBY movements can also be correspondingly classified into the nascent, developmental, and mature periods. Scholars in all periods have also presented various views on the nature of NIMBY [4].

In the nascent and developmental periods, most scholars viewed NIMBY as an unjustified emotional behavior, arguing that NIMBY movement originated from citizens' protection of their personal self-interest and was an extreme act of citizens' stubborn opposition to the construction of public facilities that they believed may adversely affect their living. For instance, Frey et al. contended that NIMBY is “beneficial for citizens but harmful to individuals” [5]. However, the viewpoint only emphasized citizens' tolerance obligation but did not take into account their environmental rights, ignoring citizens' desire and pursuit of a better environment. The deviation from understanding the nature of NIMBY directly triggered strong opposition of citizens in a community, instead culminating an extreme NIMBY movement. After the mature period, scholars reflected on the deviation of defining NIMBY In the past and redefined NIMBY from various angles. Before the environmental justice theory, scholars analyzed NIMBY in terms of social governance, economics, and psychology. Regarding social governance, when preventing and controlling social incidents, NIMBY is considered as an overreaction of citizens to influence government decisions out of their own interests, while maintaining social stability is a targeted countermeasure, ignoring the legitimate demands of citizens [6]. From the perspective of economics, the main consideration is about interest. The NIMBY phenomenon is attributed to the conflict between public interests and citizens' environmental interests, which eventually leads to the paradox of public interests and individual interests. [7] From a psychological perspective, the main focus is on the process from the formation of the NIMBY mentality to the NIMBY behavior influenced by the mentality. The behavior is simply attributed to the citizens' overreaction, which disregards the negative externalities of NIMBY facilities and presents a biased understanding of the nature of NIMBY [8].

RETRACTED

In contrast to the psychological, economic, and social governance perspectives that stigmatize NIMBY movements, such movements are perceived from the perspective of civil environmental rights to recognize citizens' environmental rights to live and develop in a beautiful comfortable environment and confront the just distribution of citizens' tolerance obligations and environmental rights. The essence of NIMBY is defined as a just movement in which citizens stand for equal environmental rights.

### 2.2. Source of Rationality of NIMBY Movements: Civil Environmental Rights

The concept of environmental rights originated in the West in the 1960s, roughly fifty years ago [9]. More than 30 years earlier, Ken.saro-Wiwa declared that “the environment (right) is the primary right of human beings” [10].

As of 2010, 142 of 198 UN member states had recognized environmental rights directly or indirectly in their constitutions, with civil and environmental laws in Germany, Russia, and Switzerland, among others, containing specific provisions for environmental rights [11]. In terms of its attributes, the right to environment is a nonproperty right related to personality, and its exercise is personality-oriented and nonproperty. In other words, the exercise of environmental rights is only based on personality needs (such as people's needs for peaceful enjoyment of health, comfort). It neither pursues the acquisition or appreciation of wealth nor consumes or costs environmental elements [12].

The basic environmental rights of citizens means that citizens enjoy the rights to live and develop in a healthy, comfortable, and beautiful environment. The rights are mainly manifested in substantive and procedural environmental rights and interests. The former includes the rights to life and health, clean air, water, light, ventilation, and peace, and the latter includes the rights to know about the government's environmental decisions and actions and make corresponding suggestions. Since citizens have the right to enjoy a good eco-environment, citizens' NIMBY movement cannot be simply categorized as an irrational act of affecting the public interest at the expense of their private interests. For the purpose of defending their legitimate rights and interests, citizens' resistance and protection measures are evidently justified when the healthy, comfortable, and beautiful environment they enjoy is affected and destroyed. Hence such a NIMBY movement is just. Of course, the basic civil environmental rights have boundaries, beyond which they fall within the category of citizens' tolerance obligations. A NIMBY movement perceptibly has its boundaries that depend on the legal boundary between civil environmental rights and tolerance obligations. Various environmental laws and regulations contain provisions regarding the scope of civil environmental rights and the degree of tolerance obligations. A NIMBY movement beyond the legal boundary may abuse basic environmental rights and violate tolerance obligations, developing into extreme environmentalism and extreme individualism and then into an obstacle to social development and public interests.

### 2.3. Analysis of the Causes of NIMBY Movement

Although the facilities that trigger a NIMBY movement are the necessities of citizens' production and life, their unique nature would inevitably lead to a NIMBY movement if citizens' legitimate environmental rights and interests are not taken into account in the site selection and construction. From the perspective of citizens' environmental rights, NIMBY movement can be attributed to the disregard to citizens' substantive and procedural environmental rights and interests.

RETRACTED

#### 2.3.1. Disregard for Substantive Environmental Rights and Interests of Citizens

The current primary and direct cause of NIMBY movements lies in the disregard for citizens' rights to clean air, water, light, ventilation, peace, and other substantive environmental rights and interests in making a decision to establish NIMBY facilities. Therefore, it is difficult for citizens to develop a corresponding sense of identity while their rights and interests are violated [13]. The scope of relevant environmental laws and regulations in China is not clearly defined regarding citizens' substantive environmental rights and interests. Although citizens are legally granted corresponding substantive environmental rights and interests, which are mostly declaratory in nature, in practice, it is difficult to identify the boundary between citizens' substantive environmental rights and interests and tolerance obligations. NIMBY facilities involve a significant derogation of civil environmental rights and interests. In this case, the government's decisions are based on ambiguous norms, directly leading to the lack of citizens' sense of identity. It is difficult for the government to meet citizens' desire for justice. The difficulty results in a de facto recognition that justice has been denied. Also, some governments are still dealing with the NIMBY problem simply as a group incident through stabilization measures. It is difficult to truly recognize the legitimate environmental rights and interests of citizens and solve the problem based on the recognition. In the case of Wuhan Yangluo waste-to-energy project, for example, the government responded to citizens' concerns about the proximity of the site to universities and communities and the impact of the odor from the dump on their living by means of an environmental impact assessment (EIA) report, ignoring the citizens' demand for clean air. This led to a large mass incident, which was followed by a simple brutal halt. According to the government, the project would not commence if the public did not agree. Such a stabilization approach has not only led to an unhealthy atmosphere of “distribution by the degree of instability,” but also greatly affected the credibility of the government.

#### 2.3.2. Disregard for Citizens' Procedural Environmental Rights and Interests

Currently, China's decision-making mechanism for NIMBY facilities is mostly a model featuring “decision-making, declaration, and defense.” The top-down model behind the scenes derives more of its advice from expert assessments. Citizens are excluded from the consultation agenda, which ignores citizens' procedural environmental rights and interests, such as the rights to know about information and make suggestions, and impedes their demands for legitimate interests.

RETRACTED

On the one hand, the current decision-making model of NIMBY facilities is more biased towards the risk value obtained by experts and scholars using statistical models. The government demonstrates the feasibility of NIMBY projects from the technical perspective, finally informing citizens of the optimal scheme obtained accordingly. According to the approach, citizens can only passively participate in and receive decisions on building NIMBY facilities, with their right to know about decisions not fully exercised. Compared with experts, laymen tend to overestimate risks, in particular when what they receive is ambiguous expertise [14]. This does not mean, however, that citizens deny the role of professional knowledge and skills in perceiving risks. What citizens oppose more is the monopoly authority of experts over risk information [15]. The current model of decision-making ignores citizens' subjective perception of risks, emphasizing the objective risk as the basis for decisions on NIMBY projects. It is difficult to convince citizens to abandon their risk perceptions based on their experiences. In the absence of communication, this situation reinforces citizens' mistrust of experts' conclusions and contributes to their resentment against the risk information monopolized by experts and scholars. Conclusions that are originally science-based become, in the eyes of the citizens, an expert's embellishment of a NIMBY project, triggering rebelliousness among citizens and intensifying a conflict between citizens and the government. Citizens' opinions and suggestions on the current decision-making model for NIMBY facilities are made late. The chain of engagement is short, with decisions made public prior to approval of site and planning and at the EIA stage. The passive and solicited nature of the engagement approach is prominent, resulting in that citizens engage in NIMBY movements due to derogated trust interests and reducing credibility of the government.

On the other hand, the existing information disclosure channels for the planning and operation of NIMBY projects are few and the public information is sketchy, resulting in that the public do not obtain project information in a timely manner or even are informed of the relevant information in a casual and passive situation. However, the preliminary work of project has been done in an orderly manner. The lack of information disclosure and transparency has become a strategic arrangement to hinder or circumvent public engagement or to propose a project site. In essence, this practice is building up conflicts for NIMBY protests. At the EIA stage, where public participation is legally required, the public in the vicinity of a NIMBY project is circumvented in selecting participants. The only channel for releasing the EIA report with citizens less informed is chosen to make the simplified version public within the shortest legal period. The practices have exacerbated public resistance to NIMBY facilities.

RETRACTED

#### 2.3.3. Analysis of the Sustainable Governance Path of NIMBY Movement

Sustainable governance is a new paradigm of governance that differs from movement-based governance. If campaign-styled governance represents an old management paradigm, sustainable governance is a new public management paradigm. The campaign-styled governance has pan-politicization thoughts, attempting to achieve change through the promotion of authority. It advocates external and imposed changes, emphasizes the rule of others, attaches importance to consistency and obedience, stresses monism and denies diversity, advocates centralization rather than sharing of power, and swings between ideal and reality [16], while sustainable governance is just the opposite, which emphasizes sharing power and responsibility and realizes sustainable public governance with the cooperation of citizen participation, social autonomy, and government governance. It emphasizes that the rule of law attaches importance to consultation in order to resolve the opposition and conflict between the government, citizens, and other stakeholders. Its focus is placed on multiagent, multi-interaction and active change; that is, governance subjects improve their governance ability through continuous learning based on the vision and purpose of improving governance performance [17]. Compared with campaign-styled governance, sustainable governance pays more attention to the environmental rights and interests of residents' entities and procedures, pays more attention to the value of democracy and rule of law, emphasizes the rule by law and public participation, and can better reflect the core interests and demands of multiple subjects. Therefore, the sustainable governance of NIMBY movements can fully respect and recognize civil environmental rights and explore effective governance of NIMBY movements within the framework of civil environmental rights.

### 2.4. Determining the Boundaries of Citizens' Substantive Environmental Rights and Interests and Enhancing Their Sense of Identity

It is difficult for citizens to develop a sense of identity for their derogated rights and interests, making it hard to recognize justice. To solve this problem, we must first define the meaning of citizens' substantive environmental rights and interests, further refine laws and regulations, determine the boundary between citizens' rights to clean air, water, light, ventilation, and peace, and clarify the boundary of citizens' tolerance obligations. On this basis, first, the government, when making decisions on NIMBY facilities, should prudently consider whether the derogation of citizens' environmental rights and interests exceeds the boundary of tolerance obligations. The government should take technical measures or reduce the scale of projects that exceed the boundary, so that the environmental burden can fall within the boundary. Second, when the government is faced with a NIMBY movement, it needs to abandon the past governance model of “maintaining the stability.” It should communicate with citizens, listen to their demands, and review the boundary of citizens' environmental rights and tolerance obligations in accordance with relevant laws and regulations. The government should respond to citizens' reasonable demands and, conversely, provide them with timely explanations. Finally, while recognizing the rationality of a NIMBY movement, the government should educate citizens about their identity. In education, it should focus on not only raising citizens' awareness of their rights, but also enhancing their awareness of responsibilities and duties. The government should build an identity education system in which rights are consistent with responsibilities, in order to teach citizens that responsibilities and duties are not the antithesis of individual rights and freedoms. The conscious performance of duties and responsibilities stems from the identification with the public value of society and the consistency of rights and obligations. This motivates citizens to spontaneously assume environmental tolerance obligations and responsibilities and fundamentally promotes a change in citizenship thinking.

RETRACTED

### 2.5. Focusing on the Sustainable Governance of NIMBY Movement and Safeguarding Citizens' Procedural Environmental Rights and Interests

The paradigm of sustainable governance calls for shared rights and joint consultation, emphasizing the rule of law and pluralistic interaction. In order to realize the sustainable governance of NIMBY movement, it is necessary to take corresponding governance instruments in the process of NIMBY decision-making at different points.

#### 2.5.1. Before NIMBY Decision-Making

Before making a decision on a NIMBY facility, first of all, the government should strengthen communication with citizens in the NIMBY area, encourage the consultation between NIMBY enterprises and citizens, and change the model featuring decision-making, declaration, and defense to one characterized by engagement, consultation, and consensus. The latter model involves the government, enterprises, and citizens in the whole process. In response to the problems of late citizen engagement, low sense of existence, and lack of ways to express demands regarding the site of NIMBY facilities, the citizen engagement chain can be lengthened to introduce the engagement and interaction of pluralistic subjects, so that multiple parties can reach a consensus on risks and benefits compensation of NIMBY facilities [18]. The consensus is reached through consultation before the decision and announcement. Then, the government and NIMBY enterprises should disclose the planning information of NIMBY projects through multiple channels to safeguard citizens' rights to know about information. Finally, in the EIA, environmental quality assessment, and social stability risk assessment, assessment subjects need to pay attention to explaining professional information to lay persons and convert terms into the expressions understood by citizens, so as to eliminate differences in citizens' risk perceptions.

#### 2.5.2. In the Construction of NIMBY Facilities

In building NIMBY facilities, both the government and the enterprises need to attach importance to disclosing construction information and maintain communication channels with citizens at the project site. NIMBY facility enterprises should timely publicize various matters concerning citizens' environmental rights and interests via various means, such as community bulletins and enterprise websites. They should communicate with citizens to resolve any inconsistencies in the plan negotiated prior to actual construction, as well as any additional derogations of citizens' environmental rights and interests due to construction and other reasons. Local governments can also work with enterprises and local citizens or village committees to set up leadership groups to deal with relevant problems promptly. The leadership group does a good job of serving as a bridge between the public, enterprises, and the government and communicates with the public to ensure that their environmental demands can be resolved.

#### 2.5.3. After the Completion of NIMBY Facilities

The completion of NIMBY facilities does not mean the end of NIMBY governance. There is still an ongoing need for regulatory revisits to NIMBY projects that have been up and running. The four types of facilities proposed by China's Ministry of Ecology and Environment cover urban sewage treatment, domestic waste treatment, treatment of hazardous refuse and waste electronic products, and environmental monitoring. They should be strictly accessible to citizens on a regular basis. NIMBY facilities should be equipped with pollutant monitoring devices by the law so as to monitor the discharge information in real time. The automatic monitoring system should be networked with the environmental department to facilitate its law enforcement and supervision, while the discharge information should be made public on time to citizens in the community where a site is located. In conclusion, the completion of NIMBY facilities is only the starting point of the governance. When the facilities are in operation, it is essential to lay more emphasis on supervising the pollutant discharge of NIMBY enterprises, increase the information disclosure of completed and operating projects, and establish a good mutual trust with neighboring citizens to avoid NIMBY incidents [19].

RETRACTED

## 3. Conclusions

As Martin Wolsink said, the stigmatization of the word “NIMBY” will hinder the analysis of the environmental interests of opponents in the NIMBY movement [19]. The word “NIMBY” is a tool to describe the reality, rather than a means of stigmatization. Simply taking the NIMBY movement as an event that destroys social stability is not only suspected of stigmatizing residents' legitimate rights protection actions, but also has the problem of endorsing the construction of illegal projects, which is not conducive to the governance of the NIMBY movement but will stimulate more and more serious social contradictions and conflicts [20]. Therefore, taking citizens' basic environmental rights as the discussion center, this paper clarifies the essence of the NIMBY movement, discusses the legitimacy of the NIMBY movement, and analyzes the causes of the NIMBY movement on the basis of correcting the names of residents who take legitimate NIMBY actions. At the same time, the governance effect of the NIMBY movement directly depends on the effectiveness of institutional arrangements and policy design formed with the joint participation of public governance subjects. Therefore, exploring the governance path of the NIMBY movement from the perspective of sustainable governance is the key to addressing the NIMBY problem and the starting point to solve the NIMBY problem.

## Data Availability

No data were used to support this study.
